# Effect of Ankle Proprioception Training on Preventing Ankle Injury of Martial Arts Athletes

This article has been retracted.

**DOI:** 10.1155/2022/8867724

**Published:** 2022-10-07

**Authors:** Ning Yu

**Affiliations:** Police Sports Department, Shaanxi Police College, Xi'an, 710021 Shaanxi, China

## Abstract

Martial arts routines originated in China and are a traditional sport of the Chinese nation. They are one of the outstanding sports culture representatives in China since ancient times. Excessively difficult movements in some martial arts routines during competitions or training can cause athlete injuries. The purpose of this article is to study the effect of proprioceptive training of ankle joints on preventing ankle injuries in martial arts athletes. Can ankle strength training and ankle proprioceptive training combined with strength training improve the dynamic and static balance of football players? This article analyzes the mechanism and causes of martial arts athletes' injuries and proposes treatment methods for ankle injuries. In the experimental part of this article, 16 martial arts athletes (8 males and 8 females) were selected as research objects, and they were randomly divided into 4 male and female experimental groups and 4 control groups. The experimental group received ankle muscle strength training for 6 weeks, and the control group received ankle muscle strength training and ankle proprioception training. The experimental results prove that ankle proprioceptive training can improve the dynamic and static balance of martial arts athletes and can effectively prevent the occurrence of ankle injury. In this paper, the dynamic balance ability in the biped standing state with eyes closed was tested, and the reductions of the stability index in the front and back directions of the control group and the experimental group were 0.03 and 0.2, respectively. It can be seen that the stability training effect of the experimental group was obvious.

## 1. Introduction

Wushu is an excellent traditional sport of the Chinese nation and an important part of China's excellent culture. Its sports characteristics determine the high requirements for the physical fitness of athletes. With the internationalization of martial arts and the requirements of new rules of martial arts and martial arts routines, the difficulty of martial arts continues to increase; martial arts sports further develops to high, difficult, floating, and stable; and the physical fitness requirements of martial arts routine athletes also increase, so the incidence of sports injuries has also increased significantly, affecting the continuity of athlete training. Ankle injury is one of the frequently occurring sports injuries in martial art routine injuries. This article explores the effects of ankle muscle strength training and proprioceptive training on the balance of the human body. It is aimed at preventing and reducing the ankle injury of martial arts athletes, laying a solid foundation for future scientific research, providing professional martial arts athletes and amateur martial arts enthusiasts, and providing scientific training basis.

Research on ankle joint, proprioceptive training, martial arts athletes, ankle joint injury, and muscle training has been ongoing. Despite extensive clinical and basic scientific research, the incidence of chronic ankle instability (CAI) has not been significantly reduced. Because the etiology of CAI is not well understood, rehabilitation treatment still faces great challenges. One of the treatments of particular concern for this injury is Kinesio Taping (KT). In this study, Kinesio Taping investigated the effect of three KT methods on the performance of CAI athletes [1]. Hunt et al.'s team believes that injury to the distal ligament of the tibia and fibula is indicative of long-term ankle dysfunction. Significant changes in ankle kinematics and contact mechanics can explain why moderate joint syndrome injuries take longer to heal and are more likely to develop long-term dysfunction and potentially cause ankle arthritis [2]. The goal of Balić et al.'s team is to evaluate the effectiveness of proprioceptive training programs based on quantifiable instability to reduce ankle sprains, knee sprains, and low back pain by developing sound and durable proprioceptive controls. 55 topics were studied. In the first biennium (2004-2006), the prevention program included classic proprioceptive exercises. In the second biennium (2006-2008), proprioceptive training became quantifiable and interactive through the electronic proprioceptive platform. In the third biennium (2008-2010), intensity and training volume increased, while training time decreased. They found that improved proprioceptive control in the single position may be a key factor in effectively reducing ankle sprains, knee sprains, and low back pain [3]. The data of this type of research has not been fully analyzed, and the real role of the data cannot be mined.

This article analyzes the mechanism and causes of martial arts athletes' injuries and then proposes a treatment method for ankle injuries. In the experimental part, 16 martial arts athletes (8 males and 8 females) were selected as research objects, and they were randomly divided into 4 male and female experimental groups and 4 control groups. The experimental group received ankle muscle strength training for 6 weeks, and the control group received ankle muscle strength training and ankle proprioception training. The experimental results prove that ankle proprioceptive training can improve the dynamic and static balance of martial arts athletes and can effectively prevent the occurrence of ankle injury.

## 2. Proposed Method

### 2.1. Proprioception of the Ankle Joint

#### 2.1.1. Proprioception

For proprioceptive sensory receptors, it is located in the skin, muscles, and joints, and the information provided by the tendons and ligaments is input to the central nervous system and is related to tissue damage [4, 5]. However, the vision and vestibular center can also send messages to maintain the balance and position of the body to the central nervous system. Therefore, trauma is likely to cause damage to the mechanoreceptors contained in the tissue and cause some tissues to lose their function and reduce the proprioceptive ability [6]. Therefore, the repeated damage to the organization is likely to be caused by the lack of feedback on proprioception. However, research shows that rehabilitation of the shoulder and knee joints after surgery can at least partially restore joint motion and joint position. For athletes who want to return to the field after an injury or after surgery, it is necessary to obtain neuromuscular control. The central nervous system integrates peripheral mechanoreceptors and vestibular and visual afferent neural signals and generates action responses. These reactions are gradually lost under three levels of motion control: spinal reflexes, cognitive coding, and brainstem activity. When the joint is under the load of mechanical force, the stability of the muscle is reflected by the stimulation of the spinal cord [7]. Cognitive coding includes the functions of the highest-order central nervous system (motor cortex, basal nucleus, and cerebellum), which are used to repeat and store autonomous actions and serve as a central nervous system command. If you are aware of your body's position and movement, you can perform various command actions without continuously giving conscious reference.

#### 2.1.2. Proprioception of the Ankle Joint

Chronic ankle instability can cause disability of the mechanoreceptors of the injured joints [8]. The ankle joint with an ankle sprain has a lower maintenance time when standing on one foot than the ankle joint with no sprain on the opposite side. Development of highly skilled systems to assess the effects of musculoskeletal injury on balance has been attempted to quantify static and dynamic proprioception. The assessment method is based on the proprioceptive sensation of the joint that is damaged after the injury, resulting in a decrease in the feedback of the lateral ligament afferent nerves and thus an increase in body swing. The impact of functionally unstable ankle joint reconstruction on proprioceptive afferent pathways has not been thoroughly studied by measuring the sensitivity or balance of joint position and body swing [9, 10]. After acute or chronic ankle injury, observation-based evidence shows that proprioceptive training techniques are very effective [11, 12].

### 2.2. Ankle Injury Analysis of Martial Arts Athletes

#### 2.2.1. Analysis of Ankle Injury Mechanism

The ankle joint is one of the more complex joints of the human body. Anatomically, the ankle joint is the part where the human foot is connected to the leg. It consists of 7 metatarsal bones plus the metatarsal bones of the foot and the bones of the lower leg [13]. The ankle supports the weight of the entire body. The ankle is composed of relatively small bones and thick and short ligaments. The main ligaments are anterior talofibular ligament, calcaneal fibula ligament, posterior talofibular ligament, and triangular ligament. The injuries are mainly valgus and varus injuries. For example, during a martial arts routine exercise, when a high-speed continuous flipping step is performed, the foot is strongly twisted to the outside and the medial ligament is stretched to cause valgus damage. Because the medial ligament is quite strong, it is often a serious injury such as a fracture or a tear. On the other hand, martial arts athletes, such as the spinner, turn 720 degrees on the ground and step on the foot because the soles are strongly twisted to the inside, and the lateral ligaments bear the load and stretch caused by varus injury [14]. In general, varus injury is more common, and eversion injury is more serious to athletes.

#### 2.2.2. Analysis of the Causes of Ankle Injury of Martial Arts Athletes

*(1) Characteristics of Wushu Sports*. The martial art routine exercise has a comprehensive requirement for speed, strength, endurance, flexibility, coordination, and sensitivity. It is a whole-body exercise that requires extreme speed. It includes speed running, flipping, turning, and sudden explosive take-off [15, 16]. The athlete's body, especially the ankle joint, causes a large load. If the ankle joint cannot withstand the load of martial arts, its load exceeds the physiological characteristics of the ankle joint, which will inevitably cause ankle injury. With the internationalization of martial arts routines and the progress of new martial arts rules, its requirements will become higher and higher. The dynamic link between movement difficulty and explosive jumping in situ increases joint stimulation. The stimulation of the joints is increased. A slight deviation of the torsion of the joints and the flashing movements in the extreme speed on the ankle joint are likely to cause ankle injury [17, 18]. At the same time, mastering such complex movements requires martial arts routine athletes to train hard day after day, resulting in long-term high load on the ankle joint, and the probability of sports injuries is further increased.

*(2) Physiological Reasons of Martial Arts Athletes*.

1. Lack of adequate preparatory activities. Before the game, because some coaches and athletes neglected the preparatory activities or just made some special preparations, ignoring the regular warm-up preparations, so the preparation activities can reduce the viscosity of the muscles and improve the excitability of the nerves. Be well prepared for the upcoming workout. The main purpose of preparation is to improve the overall metabolism of the cerebral cortex, improve its excited state, and reduce sports injuries. This activity has not started yet. If it is a simple leg press, kick, and simple jogging, it is likely to cause ankle injury
2. The physiological structure of the ankle joint is composed of the articular surface of the lower end of the tibia and fibula and the talar block, so it is also called the talar calf joint. The “sacral” joint socket formed by the lower articular surface of the tibia and the articular surfaces of the inner and outer ankles accommodates the talar block (joint head). Because the front and back of the block are wide and narrow, when the foot is dorsiflexed, the wider front part enters in the fossa; the joints are stable; however, during plantar flexion, such as when the narrow rear part of the pulley enters the fossa when walking downhill, the ankle joint is loose and can perform side movements. At this time, the ankle joint is prone to sprains and the most common varus injury. Because the lateral malleolus is longer and lower than the medial malleolus, it prevents excessive talus eversion. The martial art routine moves in a fast pace, and the load on the ankle joints, such as jumps, jumps, and landings, is large, which can cause injury if a little careless
3. Insufficient ankle joint strength, large range of martial arts sports, and long-term martial arts sports training make martial arts routine athletes' joints more flexible and more active, which reduces joint strength and stability of the joints. More so, less targeted ankle strength exercises are also the cause of ankle injury
4. The local load is too large. The swing and turn of the martial arts routine and the take-off and landing all stimulate the ankle joint. Especially, the rotation take-off and landing in the martial arts jump will increase the load on the ankle joint. The ankle load causes damage to the ankle joint

### 2.3. Treatment of Ankle Injuries

#### 2.3.1. Conventional Treatment

Conventional treatment methods are suitable for most sports injuries. The conventional treatment method for the acute stage after ankle injury is mainly to follow the “PRICE” principle, that is, first to rest and avoid weight bearing to eliminate swelling and tissue self-repair, apply ice to the affected area within 48 hours, reduce bleeding, and reduce pain and pressure bandaging, while raising the injured ankle to a higher position than the heart, in order to achieve the purpose of pain relief, swelling, and hemostasis. In more serious cases, brace fixation and other methods can be adopted, and on the basis of basic protection, go to the hospital as soon as possible to take X-rays to rule out the possibility of fractures. After the symptoms in the acute phase are basically relieved, after the pain is eliminated, traditional Chinese medical treatment and physical therapy are added, such as massage, acupuncture, electrotherapy, freezing, and manual treatment by a rehabilitation physician. Adhesion and fibrous tissue hyperplasia cause negative effects such as decreased ankle mobility.

The conventional treatment method of the ankle joint is mainly to achieve a certain degree of protection for the injured part and reduce the adverse effects caused by the injury [19]. It mainly uses the knowledge of human physiology to achieve clinical rehabilitation effects such as hemostasis, swelling, and pain relief. However, it is obviously not enough to restore normal ankle function. Necessary strength training, active joint activity exercises, and proprioception exercises need to be added to the subsequent rehabilitation.

#### 2.3.2. Muscle Training

Muscle strength training is an indispensable part in the rehabilitation training of athletes after injury. After the injury occurs, it is usually accompanied by different degrees of pain, swelling, effusion, and other symptoms. The previous treatment will generally be braked and physical therapy; until the joint range of motion is restored, the pain is reduced or even eliminated before muscle training.

The purpose of muscle strength training after ankle injury is twofold: to restore muscle dysfunction such as atrophic muscle atrophy caused by braking and reduced motion and to restore articular muscle weakness caused by ankle injury. Strengthening the muscle strength of related muscle groups around the ankle through muscle training is considered to be an important means to increase joint stability and prevent reinjury. However, for sports injuries such as ankle sprains and closed soft tissue injuries, the negative effects of ligament damage are more significant than changes in muscle function. Some studies have found that the muscle tissue around the ankle joint is not damaged, and even the muscle strength is not obviously decreased, but the function of the ankle joint was limited. Through strengthening the muscle strength of the ankle-related muscle groups, it can promote ankle rehabilitation and prevent repeated injuries. Although the muscle strength around the ankle joint has increased, the stability of the ankle joint and the risk of reinjury have not decreased. Therefore, as an exercise method commonly used for sports injuries or sports training, the role of muscle strength training in developing motor skills and improving athletic ability has been affirmed in various sports, but muscle strength training has an important role in the rehabilitation of ankle injuries. How important is the importance? The physiological mechanism of the effect of muscle training on ankle joint rehabilitation needs further research. It may be because the increase of mechanoreceptor function in muscle leads to the promotion effect of muscle training on ankle joint rehabilitation. Therefore, in terms of the current research results, it can be considered that muscle training is not the first treatment that should be considered in the early rehabilitation of ankle injury.

#### 2.3.3. Neuromuscular Control

Proprioceptive training is not a specific training method but refers to the comprehensive neuromuscular regulation of the use of different training methods to fully mobilize the body's proprioceptive sense and proprioceptors for body posture judgment, motor process perception, and motor unit activation. In the rehabilitation training after ankle sprain, many therapists will choose balance training as an important method to restore the functional neuromuscular control function of the ankle joint. After the first ankle sprain, the proprioceptors in the ankle ligament were damaged and blocked the nerve afferent pathway of motor signals. This may also explain the increased risk of repeated sprains often after ankle injury. Studies have also shown that this kind of balance training has played a significant role in preventing ankle joint instability from preventing functional ankle instability. Balance training usually requires the patient to stand on an unstable plane, such as a swing plate, foam material, or a special ankle dynamic balance trainer. It is believed that standing on an unbalanced plane can mobilize the proprioceptors around the ankle joint to participate in motion regulation, thereby conducive to the improvement of ankle joint stability. This kind of balance training has been found to be beneficial to improve the proprioception of ankle joints in different sports studies, and studies have shown that the risk of athlete reinjury has decreased.

## 3. Experiments

### 3.1. Data Collection

This article selects a total of 16 martial arts athletes, including 8 males and 8 females, and randomly divides them into 4 experimental groups and 4 control groups. The subjects were in good health and had no history of motor system, nervous system disease, or other serious diseases. There was no strenuous exercise in the day before the experiment. The athlete's nondominant leg is defined as the most commonly used support leg when shooting. All subjects' nondominant leg in this experiment is the left leg. The experimental group was mainly trained in ankle strength and proprioception, while the control group was only trained in ankle strength.

### 3.2. Experimental Methods

The experimental group received strength training around the ankle while increasing the proprioception of the ankle joint, while the control group received only strength training around the ankle. The training time is 5-8 minutes. The training time of the experimental group is slightly longer, but it will not exceed 15 minutes. It includes a series of training for ankle joints, including closed eyes, open eyes, single foot stand, and balance plate training. In addition, the same training program will be carried out after the completion of its special physical training. The basic actions of specific training are as follows:

For fibula length muscle training, an elastic band is placed on the outside of the foot to give proper tension, and then, the foot is doing valgus exercise; for tibialis anterior muscle strength training, an elastic band is placed on the instep of the foot, appropriate tension is given, and then, do toe exercise; for calf triceps strength training, stand on one foot and do heel lifting exercises; each of the above exercises is done in 2 groups; each group is done 15-20 times.

For standing with closed eyes and one foot, train 2 groups at a time; each group is performed for 30 seconds with the eyes closed, and the left and right feet are counted as one group. For standing with one foot on a balance plate, each training has 2 groups, each group is performed for 30 seconds with the eyes open, and the left and right feet are counted as a group.

### 3.3. Test Indicators

The balance ability test includes posture stability tests (open and closed eyes) and athletes' one-foot balance test.

*Posture stability test indicators*: overall stability index (SI), front-back direction stability index (A/PSI), left-right direction stability index (M/LSI), and unit: angle (°).

*One-foot balance test index*: overall stability index (SI), front-back direction stability index (A/PSI), left-right direction stability index (M/LSI), and unit: angle (°).

### 3.4. Statistics

This article uses Excel2010 to process the data before and after the experiment. Each parameter is expressed as the mean ± standard deviation. The statistical analysis is performed using SPSS18.0 software. The test method is multivariate analysis of variance and paired sample *T* test [20]. Multivariate analysis of variance means the analysis of variance of multivariate data, and it is the promotion of univariate analysis of variance. The significance level is 0.05.

## 4. Discussion

### 4.1. Analysis of the Dynamic Balance Ability with the Eyes Open and Eyes Closed

#### 4.1.1. Analysis of Dynamic Balance Ability with Both Eyes Standing

The participants were 50 males and 50 males selected from colleges and universities in City A. After three layers of selection, only 16 males and 14 females were left. Age is 18-22 years old. The overall stability index (SI) reflects the subject's overall mean swing angle or swing when standing. Anterior-posterior stability index (A/PSI) reflects the average swing angle or swing of the subject on the sagittal plane when they stand. The left and right stability index (M/LSI) reflects the average swing angle or swing of the subject on the frontal plane when standing. The lower the above value, the smaller the degree of body shaking, indicating the stronger the ability to balance. Multivariate analysis of variance was used to analyze the test results of SI, A/PSI, and M/LSI under open-eye biped standing conditions. The factors were gender (male, female), group (experimental group, control group), and test time (0 week, 6 weeks). The results showed that gender and group had no significant difference in the dynamic balance ability when standing with the eyes open and biped standing. The overall stability index (SI) and the left and right stability index (M/LSI) had significant effects before and after the test. The values of SI and M/LSI decreased significantly afterwards, with *P* values of 0.033 and 0.001, respectively. For the forward/backward direction stability index (A/PSI), the value after training has a tendency to be smaller than that before training, but there is no significant difference. The results of the test of the dynamic balance ability with the eyes and feet standing are shown in Table 1 and Figure 1.

As can be seen from Table 1 and Figure 1, for the difference of the overall stability index before and after the experiment, the change in the experimental group was significantly greater than that in the control group. The paired sample *T* test was used to compare the stability index (A/PSI) and the stability index (M/LSI) analysis and found that for standing with eyes open, the stability index before and after is significantly greater than the stability index between left and right, with a *P* value of 0.036.

#### 4.1.2. Dynamic Balance Ability with Eyes Closed and Standing on Both Feet

Multivariate analysis of variance was used to analyze the results of SI, A/PSI, and M/LSI under closed-eye biped standing status. The factors were gender (male, female), group (experimental group, control group), and test time (0 weeks, 6 weeks). The results showed that gender had no significant difference in dynamic balance ability under closed-eye biped standing status; at week 0, the experimental group and control group had no significant difference in dynamic balance ability under closed-eye biped standing status. The stability index (M/LSI) has a significant effect, with a *P* value of 0.004; that is, the stability index of the closed eyes of the experimental group after 6 weeks of training is significantly smaller than that of the control group; the stability index of the closed eyes (M/LSI) tested before and after training has a significant effect. The effect is that the value after training is significantly reduced, and the *P* value is 0.002. For SI and A/PSI, there is a trend that the value after training is smaller than before training, but there is no significant difference. There is no interaction between the factors. The test results of the dynamic balance ability with the eyes closed and standing on both feet are shown in Table 2 and Figure 2.

As can be seen from Table 2 and Figure 2, for the closed-eye left and right stability index (M/LSI), both the experimental group and the control group after testing were smaller than before testing. The closed-eye M/LSI and right single-leg M/LSI of the experimental group after proprioceptive training were reduced more than the control group that received only ankle strength training; that is, the stability of proprioceptive training was better. The paired sample *T* test was used to analyze the front-back stability index (A/PSI) and left-right stability index (M/LSI).

### 4.2. Analysis of the Dynamic Balance Ability of the Left and Right Feet with One Eye Standing

#### 4.2.1. Analysis of Dynamic Balance Ability with Left Eye and Single Foot Standing

Multivariate analysis of variance was used to analyze the test results of SI, A/PSI, and M/LSI with the left foot and one foot standing with eyes open. The factors were gender, group, and test time (0 weeks, 6 weeks). The results showed that gender, group, and test time had no significant difference in the dynamic balance ability with the left foot and one foot standing with eyes open, as shown in Table 3. The analysis of the dynamic balance ability of the left foot with one eye standing in the open state revealed that although there was no statistical difference between the factors; the values of SI, A/PSI, and M/LSI tended to decrease after 6 weeks of training. The results of the dynamic balance ability test with the left foot and one foot standing with the eyes open are shown in Table 3 and Figure 3.

From Table 3 and Figure 3, it can be seen that the change of the stability index before and after the test group is greater than the stability index of the left and right. The paired sample *T* test was used to analyze the front-back stability index and left-right stability index. When the left foot was opened with one eye, the front-back stability index was significantly larger than the left-right stability index, with a *P* value of 0.001.

#### 4.2.2. Dynamic Balance Ability with the Right Foot and One Foot Standing

Multivariate analysis of variance was used to analyze the test results of SI, A/PSI, and M/LSI with the right foot and one foot standing. The factors were gender (male, female), group (experimental group, control group), and test time (0 week, 6 weeks). The results showed that gender had no significant difference in the dynamic balance ability of the right foot with one eye standing. The group had a significant effect on the right and left stability index (M/LSI) of the right foot, with a *P* value of 0.025. The stability index (A/PSI) and right and left foot left and right stability index (M/LSI) had significant effects. The values decreased significantly after training, with *P* values of 0.050 and 0.045, respectively; there was no interaction between the factors. The results of the dynamic balance ability test with the right foot and one foot standing with the eyes open is shown in Table 4 and Figure 4.

It can be seen from Figure 4 that, for the right foot and left foot left and right stability index (M/LSI), both the experimental group and the control group after testing are smaller than before testing. In addition, the right foot and one foot M/LSI of the experimental group after proprioceptive training were reduced more than the control group that received only ankle strength training; that is, the stability of proprioceptive training was better. The paired sample *T* test was used to analyze the front-back stability index (A/PSI) and left-right stability index (M/LSI). When standing with one foot on the right foot with eyes open, the front-back stability index was significantly greater than the left-right stability index, with a *P* value of 0.001.

Chronic ankle instability is one of the most common injuries in sports medicine. Total arthroscopic anterior talofibular ligament repair has become a common procedure for the treatment of chronic lateral ankle instability. By applying the concept of enhanced recovery after surgery (ERAS) to surgery, perioperative management can be optimized and perioperative complications can be reduced.

## 5. Conclusions

1. It is experimentally obtained in this paper that ankle muscle strength training and ankle proprioception training combined with muscle strength training can improve the dynamic and static balance of football players for 6 weeks and can effectively prevent the occurrence of ankle injury
2. This experiment proves that the stability of martial arts athletes is not as good as that of left and right, and the control ability in the forward direction is worse than in the backward direction. There are a lot of movements that need to change direction from left to right and emergency stop, so there are still many injuries. The poor stability of the anterior and posterior joints is likely to cause strain on the ankle joint and talus, and injuries such as football ankles are limited. The research in this article is limited. The issue of how to prevent other injuries can be studied in the future
3. The method adopted in this article is simple and easy, consumes short time, does not affect the progress of normal class hours and training time, and is suitable for promotion among school football and amateurs and football players. It is necessary to raise awareness of injury prevention and prevent it before it happens. The prevention of ankle injury should be grasped from early to enhance joint strength and cooperate with proprioceptive training

## Figures and Tables

**Figure 1:** Test results of dynamic balance ability with eyes open and standing on both feet.

**Figure 2:** Test results of dynamic balance ability with eyes closed and standing on both feet.

**Figure 3:** Test results of dynamic balance ability with the left foot and one foot standing with eyes open.

**Figure 4:** Test results of the dynamic balance ability with the right foot and one foot standing.

**Table 1:** Test results of dynamic balance ability with eyes open and standing on both feet.

Sex	Index	Test group		Control group	
		Before	After	Before	After
Male	SI	0.25	0.15	0.35	0.25
	A/PSI	0.2	0.1	0.25	0.21
	M/LSI	0.12	0.1	0.15	0.11

Female	SI	0.45	0.3	0.26	0.2
	A/PSI	0.35	0.25	0.25	0.21
	M/LSI	0.2	0.1	0.15	0.1

**Table 2:** Test results of dynamic balance ability with eyes closed and standing on both feet.

Sex	Index	Test group		Control group	
		Before	After	Before	After
Male	SI	0.75	0.5	0.9	0.8
	A/PSI	0.53	0.31	0.59	0.53
	M/LSI	0.31	0.15	0.51	0.39

Female	SI	0.89	0.71	0.69	0.57
	A/PSI	0.61	0.43	0.39	0.37
	M/LSI	0.43	0.21	0.45	0.33

**Table 3:** Test results of dynamic balance ability with left eye and one foot standing.

Sex	Index	Test group		Control group	
		Before	After	Before	After
Male	SI	0.93	0.57	0.97	0.89
	A/PSI	0.85	0.61	0.81	0.79
	M/LSI	0.65	0.51	0.59	0.51

Female	SI	0.83	0.67	1.03	0.87
	A/PSI	0.69	0.57	0.79	0.67
	M/LSI	0.49	0.35	0.59	0.43

**Table 4:** Test results of dynamic balance ability with the right foot and one foot standing.

Sex	Index	Test group		Control group	
		Before	After	Before	After
Male	SI	0.69	0.53	0.95	0.79
	A/PSI	0.63	0.47	0.71	0.63
	M/LSI	0.39	0.21	0.47	0.37

Female	SI	0.83	0.63	0.83	0.69
	A/PSI	0.65	0.47	0.69	0.61
	M/LSI	0.43	0.19	0.57	0.47

## Data Availability

No data were used to support this study.

## References

[1] Matthews J. J., Nicholas C. (2017). Extreme rapid weight loss and rapid weight gain observed in UK mixed martial arts athletes preparing for competition. *International Journal of Sport Nutrition and Exercise Metabolism*.

[2] Hunt K. J., Goeb Y., Behn A. W., Criswell B., Chou L. (2015). Ankle joint contact loads and displacement with progressive syndesmotic injury. *Foot & Ankle International*.

[3] Balić A., Bukvić Mokos Z., Marinović B., Ledić Drvar D. (2018). Tatami mats: a source of pitted keratolysis in a martial arts athlete?. *Acta Dermatovenerologica Croatica: ADC*.

[4] Dubnov-Raz G., Mashiach-Arazi Y., Nouriel A., Raz R., Constantini N. W. (2015). Can height categories replace weight categories in striking martial arts competitions? A pilot study. *Journal of Human Kinetics*.

[5] Coswig V. S., Ramos S. d. P., Del Vecchio F. B. (2016). Time-motion and biological responses in simulated mixed martial arts sparring matches. *Journal of Strength & Conditioning Research*.

[6] Xu Y., Zhu Y., Xu X.-Y. (2017). Ankle joint distraction arthroplasty for severe ankle arthritis. *BMC Musculoskeletal Disorders*.

[7] Walter W. R., Hirschmann A., Alaia E. F., Garwood E. R., Rosenberg Z. S. (2018). Journal Club: MRI evaluation of midtarsal (Chopart) sprain in the setting of acute ankle injury. *AJR: American Journal of Roentgenology: Including Diagnostic Radiology, Radiation Oncology, Nuclear Medicine, Ultrasonography and Related Basic Sciences*.

[8] Kern A. M., Anderson D. D. (2015). Expedited patient-specific assessment of contact stress exposure in the ankle joint following definitive articular fracture reduction. *Journal of Biomechanics*.

[9] Srettabunjong S. (2019). Fatal massive pulmonary embolism following a minor ankle injury as a rare cause of sudden unexpected death: a case report. *The Journal of Foot and Ankle Surgery*.

[10] Acosta-Olivo C., Tamez-Mata Y., Elizondo-Rodriguez J., Rodriguez-Torres R., Diaz-Valadez A., Peña-Martinez V. (2019). Investigation of the association between the acute ankle injury caused by fall from own height and body mass index. *The Journal of Foot and Ankle Surgery*.

[11] Kobayashi T., Watanabe K., Teramoto A., Suzuki D., Fujimiya M., Yamashita T. (2020). Biomechanical analysis of midfoot instability after bifurcate ligament injury and ankle brace application: a cadaveric study. *The Journal of Foot and Ankle Surgery*.

[12] Hartley E. M., Hoch M. C., Boling M. C. (2018). Y-balance test performance and BMI are associated with ankle sprain injury in collegiate male athletes. *Journal of Science and Medicine in Sport*.

[13] Klos K., Simons P., Mückley T., Karich B., Randt T., Knobe M. (2017). Frakturen des oberen sprunggelenks beim älteren patienten. *Der Unfallchirurg*.

[14] Riva D., Bianchi R., Rocca F., Mamo C. (2016). Proprioceptive training and injury prevention in a professional men's basketball team. *Journal of Strength & Conditioning Research*.

[15] Kim B. R., Lee H. J. (2017). Effects of proprioceptive neuromuscular facilitation-based abdominal muscle strengthening training on pulmonary function, pain, and functional disability index in chronic low back pain patients. *Journal of Exercise Rehabilitation*.

[16] Park H. R., Lee M. K., Yun T. W. (2015). Effect of proprioceptive neuromuscular facilitation and action observation training on upper extremity motor function in stroke patient: a single-subject study. *Physical Therapy Korea*.

[17] Ronga I., Franza M., Sarasso P., Neppi-Modona M. (2017). Oculomotor prismatic training is effective in ameliorating spatial neglect: a pilot study. *Experimental Brain Research*.

[18] Abdelaziz A., Mahmoud A. N. (2021). Intelligent system for forecasting failure of agile projects. *Journal of Intelligent Systems and Internet of Things*.

[19] Biz C., Nicoletti P., Tomasin M., Bragazzi N. L., Di Rubbo G., Ruggieri P. (2022). Is kinesio taping effective for sport performance and ankle function of athletes with chronic ankle instability (CAI)? A systematic review and meta-analysis. *Medicina (Kaunas, Lithuania)*.

[20] Miari M., Anan M. T., Zeina M. B. (2022). Neutrosophic two way ANOVA. *International Journal of Neutrosophic Science*.

